The article "MicroRNA-182 downregulates Wnt/β-catenin signaling, inhibits proliferation, and promotes apoptosis in human osteosarcoma cells by targeting HOXA9" was retracted in 2022. Reasons: fabricated or falsified data; manipulated images; an official misconduct investigation; misconduct by an author.

# MicroRNA-182 downregulates Wnt/β-catenin signaling, inhibits proliferation, and promotes apoptosis in human osteosarcoma cells by targeting HOXA9

**DOI:** 10.18632/oncotarget.21167

**Published:** 2017-09-22

**Authors:** Zi-Feng Zhang, Yong-Jian Wang, Shao-Hua Fan, Shi-Xin Du, Xue-Dong Li, Dong-Mei Wu, Jun Lu, Yuan-Lin Zheng

**Affiliations:** ^1^ Key Laboratory for Biotechnology on Medicinal Plants of Jiangsu Province, School of Life Science, Jiangsu Normal University, Xuzhou 221116, P.R. China; ^2^ Department of Orthopedics, The Third Affiliated Hospital, Shenzhen University, Shenzhen 518002, P.R. China

**Keywords:** microRNA-182, homeobox A9, wingless-type/β-catenin signaling pathway, osteosarcoma

## Abstract

We investigated the mechanisms by which microRNA (miR)-182 promotes apoptosis and inhibits proliferation in human osteosarcoma (OS) cells. Levels of miR-182 and Homeobox A9 (HOXA9) expression were compared between human OS and normal cells. Subjects were divided into OS and normal groups. We analyzed the target relationship of miR-182 and Homeobox A9 (HOXA9). Cells were then assigned into blank, negative control, miR-182 mimics, miR-182 inhibitors, siRNA-HOXA9, or and miR-182 inhibitors + siRNA-HOXA9 groups. Cell function was assayed by CCK-8, flow cytometry and wound healing assay. Additionally, we analyzed OS tumor growth in a xenograft mouse model. Dual-luciferase reporter assays indicated miR-182 directly targets HOXA9. Reverse transcription quantitative PCR and western blotting revealed elevated expression of miR-182, WIF-1, BIM, and Bax, and reduced expression of HOXA9, Wnt, β-catenin, Survivin, Cyclin D1, c-Myc, Mcl-1, Bcl-xL, and Snail in osteosarcoma cells treated with miR-182 mimic or siRNA-HOXA9 as compared to controls. Osteosarcoma cells also exhibited decreased cell proliferation, migration, and tumor growth, and increased apoptosis when treated with miR-182 mimic or siRNA-HOXA9. Correspondingly, in a xenograft mouse model, osteosarcoma tumor volume and growth were increased when cells were treated with miR-182 inhibitor and decreased by miR-182 mimic or siRNA-HOXA9. These results indicate that miR-182 downregulates Wnt/β-catenin signaling, inhibits cell proliferation, and promotes apoptosis in osteosarcoma cells by suppressing HOXA9 expression.

## INTRODUCTION

Osteosarcoma (OS) is the most common primary bone tumor in children. There are limited treatments and the prognosis of patients with metastatic OS is poor [1]. OS arises from primitive bone-forming mesenchymal cells. The incidence rates are 3.5–4.6 per million in children aged 0–14 years and 4.6–5.6 in children aged 0–19 years each year [2]. The molecular mechanisms underlying OS recurrence and metastasis have not been elucidated [3]. MicroRNAs (miRs) are non-coding RNAs that negatively regulate gene expression at the post-transcriptional level. Differential expression of 177 miRs was reported in 19 human OS cell lines [4]. The Wnt/β-catenin pathway has been shown to play a role in skeletal development and the specification of the osteoblast lineage and may have a key role in OS [5].

The article "MicroRNA-182 downregulates Wnt/β-catenin signaling, inhibits proliferation, and promotes apoptosis in human osteosarcoma cells by targeting HOXA9" was retracted in 2022. Reasons: fabricated or falsified data; manipulated images; an official misconduct investigation; misconduct by an author.

MiR-182, a member of the miR-183 cluster, is located on human chromosome 7q32. It is differentially expressed in various cancers [6]. Downregulation of miR-182 in OS cells enhanced tumor growth, migration, and invasion by targeting TIAM1, indicating that miR-182 may act as a tumor suppressor in OS [7]. The Wnt family consists of more than 19 secreted cysteine-rich glycoproteins. Overexpression of Wnt/β-catenin signaling proteins can promote tumor development and progression [8]. β-catenin is a multifunctional component of the Wnt/β-catenin signaling pathway that can promote both tumor cell proliferation and apoptosis in various cancers including OS [9, 10]. Wnt/β-catenin signaling is essential for embryonic development in vertebrates and patterning in invertebrates. Deregulation of Wnt/β-catenin signaling has been associated with cancer development [11, 12]. Wnt/β-catenin signaling regulates cell proliferation, differentiation, apoptosis, and migration [13, 14]. Previous studies have demonstrated that *Wnt5a/7a* overexpression promotes tumor cell senescence via the canonical Wnt/β-catenin signaling pathway [15, 16]. The Homeobox A9 (*HOXA9*) gene encodes a transcription factor that regulates embryonic development. Aberrant activation of *HOXA9* was demonstrated in glioblastoma [17]. Deregulation of *HOXA9* was also frequently observed in acute leukemias and was shown to be indispensable for hematopoietic stem cell expansion [18, 19]. Deregulated expression of HOX genes such as *HOXA9* has been associated with myeloproliferative disorders [20]. Interestingly, Wnt/β-catenin signaling was linked to *HOXA2* in mouse embryonic development [21]. Here, we investigated the mechanisms by which miR-182 inhibits proliferation and promotes apoptosis in human OS cells.

## RESULTS

### HOXA9 is upregulated in OS compared to normal tissue

We analyzed HOXA9 expression in human OS compared to normal tissue by immunohistochemistry. Cells that exhibited brown/yellow cytoplasmic staining were classified as HOXA9-positive. The positive expression rate of HOXA9 was 65.22% in OS tissue compared to 13.04% in normal tissue (*P* < 0.05) (Figure 1).

**Figure 1:** Immunohistochemical analysis of HOXA9 expression in OS compared to normal tissue (**A**) Normal tissue; (**B**) OS tissue. ^*^P < 0.05.

The article "MicroRNA-182 downregulates Wnt/β-catenin signaling, inhibits proliferation, and promotes apoptosis in human osteosarcoma cells by targeting HOXA9" was retracted in 2022. Reasons: fabricated or falsified data; manipulated images; an official misconduct investigation; misconduct by an author.

### Expression of miR-182, *HOXA9*, Wnt/β-catenin signaling pathway-, proliferation-, and apoptosis-related genes in OS compared to normal tissue

Reverse transcription quantitative PCR (RT-qPCR) analysis demonstrated that miR-182 expression as well as *WIF-1*, *BIM*, and *Bax* mRNA expression were reduced in OS compared to normal tissue. In contrast, *HOXA9*, *Survivin*, *Cyclin D1*, *c-Myc*, *Mcl-1*, *Bcl-xL*, and *Snail* mRNA expression were elevated in the OS compared to normal groups (all *P* < 0.05) (Figure 2). No differences in *Wnt* and β-catenin mRNA expression were observed between OS and normal tissue (all *P* > 0.05).

**Figure 2:** RT-qPCR analysis of miR-182, WIF-1, BIM, Bax, HOXA9, Wnt, β-catenin, Survivin, Cyclin D1, c-Myc, Mcl-1, Bcl-xL, and Snail expression in OS compared to normal tissue ^*^P < 0.05.

### Expression of HOXA9, Wnt/β-catenin signaling pathway-, proliferation-, and apoptosis-related proteins in OS and normal tissue

WIF-1, BIM, and Bax protein expression were reduced in OS compared to normal tissue (*P* < 0.05), while HOXA9, Wnt, β-catenin, Survivin, Cyclin D1, c-Myc, Mcl-1, Bcl-xL, and Snail expression was elevated in OS compared to normal tissue (*P* < 0.05) (Figure 3). MiR-182 and HOXA9 expression were elevated in OS compared to normal tissue, indicating there could be a functional connection between miR-182 and HOXA9 in OS (Figures 2 and 3). WIF-1 expression was reduced while β-catenin protein expression was elevated in OS compared to normal tissue. No differences in Wnt and β-catenin expression were observed between OS and normal tissue, indicating that Wnt/β-catenin signaling was activated in OS cells through inhibition of WIF-1 protein expression. Following activation of Wnt signaling, β-catenin enters the nucleus and complexes with T cell factor (TCF) to regulate proliferation, migration, and apoptosis in OS cells. The mRNA and protein expression of cell proliferation-related genes (*Survivin*, *c-Myc*, and *Cyclin D1*) were elevated in OS compared to normal tissue, while the levels of apoptosis-related genes (*BIM*, *Bax*, *Mcl-1*, and *Bcl-xL*) were reduced. These results indicated that caspase-induced apoptosis was inhibited in OS. Alterations in the expression of these proteins may promote OS cell migration.

**Figure 3:** Western blot analysis of WIF-1, BIM, Bax, HOXA9, Wnt, β-catenin, Survivin, Cyclin D1, c-Myc, Mcl-1, Bcl-xL, and Snail expression in OS compared to normal tissue (**A**) Histogram showing the relative expression of WIF-1, BIM, Bax, HOXA9, Wnt, β-catenin, Survivin, Cyclin D1, c-Myc, Mcl-1, Bcl-xL, and Snail in OS compared to normal tissue; (**B**) Western blot images of protein expression in OS compared to normal tissue; ^*^P < 0.05.

The article "MicroRNA-182 downregulates Wnt/β-catenin signaling, inhibits proliferation, and promotes apoptosis in human osteosarcoma cells by targeting HOXA9" was retracted in 2022. Reasons: fabricated or falsified data; manipulated images; an official misconduct investigation; misconduct by an author.

### MiR-182 expression is higher in U-2OS cells compared to other OS cell lines

We analyzed miR-182 expression in three OS cell lines (SOSP-9607, U-2OS, and MG63) by RT-qPCR (Figure 4). MiR-192 expression was highest in U-2OS cells (*P* < 0.05). Therefore, these cells were selected for the following experiments.

**Figure 4:** MiR-182 expression in SOSP-9607, U-2OS, and MG63 cells ^*^P < 0.05, compared to SOSP-9607 cells; ^#^*P* < 0.05, compared to MG63 cells.

### HOXA9 is a target of miR-182

MiR-182 has a predicted *HOXA9* binding site located in the 3′ untranslated region (3′UTR) (Figure 5A). We found that relative luciferase activity in OS cells transfected with a wild-type *HOXA9* construct (HOXA9-wt) was reduced in the miR-182 mimic compared to negative control (NC) group (*P* < 0.05). There was no difference in relative luciferase activity in OS cells transfected with a mutant *HOXA9* (HOXA9-mut) between the miR-182 mimic and NC groups (*P* > 0.05) (Figure 5B). These results demonstrated that *HOXA9* expression was negatively regulated by miR-182.

**Figure 5:** HOXA9 is a target of miR-182 (**A**) Predicted binding site of miR-182 in the *HOXA9* 3′UTR; (**B**) Comparison of luciferase activity in the NC and miR-182 mimic groups; ^*^P < 0.05, compared to the NC group.

### Expression of miR-182, *HOXA9*, Wnt/β-catenin pathway-, proliferation-, and apoptosis-related genes in OS cells following transfection

We analyzed miR-182, *WIF-1*, β-catenin, *BIM*, *Bax*, *HOXA9*, *Survivin*, *Cyclin D1*, *c-Myc*, *Mcl-1*, *Bcl-xL*, and *Snail* mRNA expression using RT-qPCR (Figure 6). Increased *WIF-1*, *BIM*, and *Bax* mRNA expression, and decreased *HOXA9*, *Wnt*, β-catenin, *Survivin*, *Cyclin D1*, *c-Myc*, *Mcl-1*, *Bcl-xL*, and *Snail* mRNA expression (all *P* < 0.05) were observed in the miR-182 mimic and siRNA-HOXA9 groups compared to blank and NC groups. No differences in the levels of these mRNAs were detected between the blank and NC groups (*P* > 0.05). MiR-182 mRNA expression was elevated in the miR-182 mimic group (*P* < 0.05). No differences in miR-182 mRNA expression were observed between the siRNA-HOXA9 and NC groups (*P* > 0.05). Reduced miR-182, *WIF-1*, *BIM*, and *Bax* expression, but elevated *HOXA9*, *Wnt*, β-catenin, *Survivin*, *Cyclin D1*, *c-Myc*, *Mcl-1*, *Bcl-xL*, and *Snail* mRNA expression was observed in the miR-182 inhibitor group (all *P* < 0.05). MiR-182 mRNA expression was reduced in the miR-182 inhibitor + siRNA-HOXA9 compared to the blank and NC groups (*P* < 0.05). No differences were observed in *HOXA9*, *Wnt*, β-catenin, *WIF-1*, *Survivin*, *Cyclin D1*, *c-Myc*, *BIM*, *Bax*, *Mcl-1*, *Bcl-xL*, and *Snail* mRNA expression between the miR-182 inhibitor + siRNA-HOXA9, blank, and NC groups (*P* > 0.05). Additionally, there were no differences in β-catenin mRNA expression between the six groups (*P* < 0.05).

The article "MicroRNA-182 downregulates Wnt/β-catenin signaling, inhibits proliferation, and promotes apoptosis in human osteosarcoma cells by targeting HOXA9" was retracted in 2022. Reasons: fabricated or falsified data; manipulated images; an official misconduct investigation; misconduct by an author.

**Figure 6:** RT-qPCR analysis of miR-182, WIF-1, β-catenin, BIM, Bax, HOXA9, Survivin, Cyclin D1, c-Myc, Mcl-1, Bcl-xL, and Snail expression following transfection (**A**) Histograms showing the relative expression of miR-182, *HOXA9*, β-catenin, and *WIF-1* in the six groups; (**B**) Histograms showing the relative expression of *Survivin*, *c-Myc*, *Cyclin D1*, and *Snail* in the six groups; (**C**) Histograms showing the relative expression of *BIM*, *Mcl-1*, *Bcl-xL*, and *Bax* in the six groups. ^*^P < 0.05, compared to the NC group.

### Expression of HOXA9, Wnt/β-catenin pathway-, proliferation-, and apoptosis-related proteins following cell transfection

We analyzed the expression of HOXA9, Wnt/β-catenin pathway-related proteins, as well as proliferation- and apoptosis-related proteins by western blotting (Figure 7). An increase in WIF-1, BIM, and Bax protein expression, and a decrease in HOXA9, Wnt, β-catenin, Survivin, Cyclin D1, c-Myc, Mcl-1, Bcl-xL, and Snail expression was observed in the miR-182 mimic and siRNA-HOXA9 groups compared to blank and NC groups. Opposite results were observed in the miR-182 inhibitor group (*P* < 0.05). There were no differences in the expression of these proteins between the blank and NC groups (*P* > 0.05). Opposite results were observed in the miR-182 inhibitor + siRNA-HOXA9 group compared to the miR-182 mimic and the miR-182 inhibitor groups.

**Figure 7:** Western blot analysis of WIF-1, BIM, Bax, HOXA9, β-catenin, Survivin, Cyclin D1, c-Myc, Mcl-1, Bcl-xL, and Snail expression in each group following transfection (**A**) Western blot images for all proteins evaluated; (**B**) Histograms showing the relative expression of HOXA9, WIF-1, and β-catenin in the six groups; (**C**) Histograms showing the relative expression of c-Myc, Survivin, Snail, and Cyclin D1 in the six groups; (**D**) Histograms showing the relative expression of BIM, Mcl-1, Bcl-xL, and Bax in the six groups; ^*^P < 0.05, compared to the NC group.

Low miR-182 expression was associated with elevated *HOXA9* expression and reduced WIF-1 expression. WIF-1 expression was elevated in the shRNA-HOXA9 group, indicating that miR-182 might regulate WIF-1 expression by directly suppressing *HOXA9* expression (Figures 6 and 7). Wnt/β-catenin signaling is activated in OS through inhibition of WIF-1 protein expression. This results in β-catenin translocation to the nucleus where it complexes with TCF to regulate proliferation, apoptosis, and migration. We also found the responses of proliferation-related genes (*Survivin*, *c-Myc*, and *Cyclin D1*), apoptosis-related genes (*BIM*, *Bax*, *Mcl-1*, and *Bcl-xL*), and the migration-related gene *Snail* to changes in β-catenin, WIF-1, and HOXA9 expression were indirectly regulated by miR-182. Opposite results were observed in the miR-182 mimic compared to miR-182 inhibitor group. Additionally, opposite results were observed in the miR-182 inhibitor + siRNA-HOXA9 group compared to the miR-182 mimic and miR-182 inhibitor groups. Our data indicate that miR-182 indirectly regulates Wnt/β-catenin signaling by decreasing *HOXA9* expression in OS.

The article "MicroRNA-182 downregulates Wnt/β-catenin signaling, inhibits proliferation, and promotes apoptosis in human osteosarcoma cells by targeting HOXA9" was retracted in 2022. Reasons: fabricated or falsified data; manipulated images; an official misconduct investigation; misconduct by an author.

### Upregulation of miR-182 and downregulation of HOXA9 inhibited U-2OS and hFOB cell proliferation

Decreased cell proliferation was observed in the miR-182 mimic and siRNA-HOXA9 groups compared to the blank and NC groups (*P* < 0.05). Increased proliferation was observed in the miR-182 inhibitor group compared to the blank and NC groups (*P* < 0.05). No differences in U-2OS and hFOB cell proliferation were observed between the blank and NC groups (*P* > 0.05). An opposite trend was observed in the miR-182 inhibitor + siRNA-HOXA9 group compared to the miR-182 mimic and miR-182 inhibitor groups (Figure 8). These data indicated that miR-182 upregulation and *HOXA9* silencing reduced the proliferation of U-2OS and hFOB cell lines *in vitro*.

**Figure 8:** CCK-8 assays to analyze differences in cell proliferation between the six groups

### Analysis of cell cycle progression and apoptosis in hFOB and U-2OS cells after transfection

We analyzed cell cycle changes in hFOB and U-2OS cells using propidium iodide (PI) staining (Figure 9). An increase in the number of cells in G0/G1 and a decrease in the number of cells in S phase were observed in the miR-182 mimic and siRNA-HOXA9 groups compared to blank and NC groups, which was indicative of inhibition of OS cell proliferation (*P* < 0.05). A decrease in the number of cells in GO/G1, and an increase in the number of cells in S phase was observed in; the miR-182 inhibitor group compared to the blank and NC control groups (*P* < 0.05). No differences in cell cycle phase were observed between the blank and NC groups (*P* > 0.05). Opposite results were observed in the miR-182 inhibitor + siRNA-HOXA9 group compared to the miR-182 mimic and miR-182 inhibitor groups.

**Figure 9:** PI staining to analyze differences in cell cycle progression between the six groups (**A**) Images showing differences in cell cycle phase in hFOB cells between the six groups; (**B**) Percentage of hFOB cells in the indicated cell cycle phases among the six groups; (**C**) Images showing differences in cell cycle phase in U-2OS cells between the six groups; (**D**) Percentage of U-2OS cells in the indicated cell cycle phases among the six groups; ^*^P < 0.05, compared to the blank and NC groups.

The article "MicroRNA-182 downregulates Wnt/β-catenin signaling, inhibits proliferation, and promotes apoptosis in human osteosarcoma cells by targeting HOXA9" was retracted in 2022. Reasons: fabricated or falsified data; manipulated images; an official misconduct investigation; misconduct by an author.

Dual Annexin-V/PI staining was used to detect apoptosis in hFOB and U-2OS cells (Figure 10). No differences in apoptosis were observed between the blank and NC groups (*P* > 0.05). A decrease in apoptosis was observed in the miR-182 mimic and siRNA-HOXA9 groups compared to the blank and NC groups (*P* < 0.05). An increase in apoptosis was observed in the miR-182 inhibitor compared to the blank and NC groups (*P* < 0.05). Opposite results were observed in the miR-182 inhibitor + siRNA-HOXA9 group compared to the miR-182 mimic and miR-182 inhibitor groups.

**Figure 10:** Annexin-V/PI staining to analyze apoptosis in OS cells (**A**) Analysis of apoptosis in hFOB cells; (**B**) Differences in the percentage of apoptotic hFOB cells between the six groups; (**C**) Analysis of apoptosis in U-2OS cells; (**D**) Differences in the percentage of apoptotic U-2OS cells between the six groups; ^*^P < 0.05, compared to the blank and NC groups.

### Analysis of hFOB and U-2OS cell migration following transfection

Inhibition of miR-182 in hFOB and U-2OS cells enhanced migration in wound healing assays compared to the blank and NC groups (*P* < 0.05). In contrast, decreased migration was observed in the miR-182 mimic and siRNA-HOXA9 groups compared to blank and NC groups (*P* < 0.05) (Figure 11). Opposite effects were observed in the miR-182 inhibitor + siRNA-HOXA9 group compared to the miR-182 mimic and miR-182 inhibitor groups.

**Figure 11:** Analysis of cell migration using wound healing assays (**A**) Images comparing cell migration in hFOB and U-2OS cells between the six groups; (**B**) Comparison of wound closure in hFOB and U-2OS cells between the six groups; wound closure: (distance_0 h_ – distance_48 h_)/distance_0 h_; ^*^P < 0.05, compared to the blank and NC groups.

### Analysis of xenograft tumor growth in nude mice

Tumor volume and growth were increased in the miR-182 inhibitor group compared to blank and NC groups (*P* < 0.05). Decreased tumor volume and growth were observed in the miR-182 mimic and siRNA-HOXA9 groups compared to blank and NC groups (*P* < 0.05). No differences in xenograft tumor volume or growth were observed between the miR-182 mimic and siRNA-HOXA9 groups compared to the blank and NC groups (*P* > 0.05) (Figure 12).

**Figure 12:** Comparison of xenograft tumor size and growth rates in the six groups (**A**) Cell growth; (**B**) Tumor size; (**C**) Western blot analysis of HOXA9, WIF-1, and β-catenin protein expression in the six groups; (**D**) Histograms showing the relative expression of HOXA9, WIF-1, and β-catenin in tumor tissue from nude mice in the six experimental groups; (**E**) Histograms showing the relative expression of c-Myc, Survivin, Snail, and Cyclin D1 in tumor tissue from mice in the six groups; (**F**) Histograms showing the relative expression of BIM, Mcl-1, Bcl-xL, and Bax in tumor tissue from mice in the six groups; ^*^P < 0.05, compared to the blank and NC groups.

The article "MicroRNA-182 downregulates Wnt/β-catenin signaling, inhibits proliferation, and promotes apoptosis in human osteosarcoma cells by targeting HOXA9" was retracted in 2022. Reasons: fabricated or falsified data; manipulated images; an official misconduct investigation; misconduct by an author.

No differences in HOXA9, WIF-1, BIM, β-catenin, Survivin, Cyclin D1, c-Myc, Bax, Mcl-1, Bcl-xL, and Snail protein expression in U-2OS cells were observed between the blank and NC groups (*P* > 0.05). An increase in WIF-1, BIM, and Bax, and a decrease in HOXA9, β-catenin, Survivin, Cyclin D1, c-Myc, Bax, Mcl-1, Bcl-xL, and Snail protein expression was observed in the miR-182 mimic and siRNA-HOXA9 groups compared to the blank and NC groups (all *P* < 0.05). In contrast, a decrease in WIF-1, BIM, and Bax, and in increase in HOXA9, β-catenin, Survivin, Cyclin D1, c-Myc, Bax, Mcl-1, Bcl-xL, and Snail protein expression were observed in the miR-182 inhibitor group compared to the blank and NC groups (all *P* < 0.05). Opposite trends in protein expression were observed in the miR-182 inhibitor + siRNA-HOXA9 group compared to the miR-182 mimic and miR-182 inhibitor groups.

## DISCUSSION

OS treatment frequently fails as a result of chemoresistance, but the mechanisms underlying drug resistance have not been fully elucidated [22]. Aberrant activation of Wnt/β-catenin signaling has been associated with local invasion, early metastasis, and relapse in OS [23, 24]. A miRNA signature associated with OS pathogenesis and progression was identified previously [25]. In this study, we investigated the mechanisms by which miR-182 inhibits cell proliferation and promotes apoptosis in OS.

We observed increased *HOXA9* expression and decreased miR-182 expression in OS compared to normal tissue. MiRNAs are non-coding RNAs that regulate gene expression at the post-transcriptional level [26]. MiR-182 has an important role in regulating cancer progression [27]. Low miR-183 expression was observed in lung cancer [28]. It was also found to be downregulated in human gastric adenocarcinoma. MiR-182 overexpression suppressed colony formation and proliferation in gastric cancer cells, suggesting that it inhibits tumor progression in gastric cancer [29]. Aberrant expression of Hox genes has been associated with tumorigenesis, suggesting that altered expression could be important for both tumor suppression and oncogenesis [30]. *HOXA9* plays a key role in both development and hematopoiesis [31, 32]. Overexpression of *HOXA9* has been observed in 70% of patients with acute myeloid leukemia (AML) [33]. Additionally, *HOXA9* overexpression has been reported in approximately 50% of AML patients and was correlated with poor prognosis [34]. Decreased *HOXA9* mRNA and protein expression were observed in the miR-182 mimic and siRNA-HOXA9 groups following transfection, indicating the miR-182 mimic and siRNA-HOXA9 had similar effects and could prevent OS progression.

The article "MicroRNA-182 downregulates Wnt/β-catenin signaling, inhibits proliferation, and promotes apoptosis in human osteosarcoma cells by targeting HOXA9" was retracted in 2022. Reasons: fabricated or falsified data; manipulated images; an official misconduct investigation; misconduct by an author.

Following transfection, increased WIF-1, BIM, and Bax expression, and decreased Wnt, β-catenin, Survivin, Cyclin D1, c-Myc, Mcl-1, Bcl-xL, and Snail expression were observed in the miR-182 mimic and siRNA-HOXA9 groups compared to the blank, NC, and miR-182 inhibitor + siRNA-HOXA9 groups. Opposite results were observed in the miR-182 inhibitor group. Bax and Bak are pro-apoptotic proteins, while Bcl-2, Bcl-xL, and Mcl-1 are anti-apoptotic [35]. Activation of Bax and Bak does not occur if all anti-apoptotic Bcl-2 proteins are neutralized [36]. BIM and Bax are apoptosis-related proteins that are targets of FOXO1, which is negatively regulated by miR-182 in response to oxidative stress [37]. Bcl-2 family members such as BIM may contribute to programmed cell death by inducing cytochrome C release from the mitochondria and activation of caspase-3 and caspase-9 [38]. Repression of the atypical Bcl-2 family member, Bcl2-like12 (Bcl2L12), was critical for miR-182 anti-tumor activity and enhanced therapeutic susceptibility [39]. Inhibition of c-Myc, cyclin D1, and Survivin, which promote tumor invasion and angiogenesis and inhibit apoptosis may be effective for the treatment of colon cancer [40]. Additionally, STAT3 suppression results in inhibition of cell survival-related proteins (Bcl-xL, Bcl-2, Survivin, Mcl-1, and cIAP-2) and proliferation (c-Myc and Cyclin D1), indicating STAT3 may be an effective therapeutic target [41]. MiR-182, a p53-dependent miRNA, was shown to inhibit *MITF*, *Bcl2*, and *Cyclin D2* expression in uveal melanoma cells, suggesting it functions as a tumor suppressor [42]. WIF-1, a negative regulator of Wnt/β-catenin signaling, has been implicated in tumorigenesis [43]. Overexpression of the miR-182/miR-183/miR-96 cluster was associated with activation of Wnt/β-catenin signaling in medulloblastoma [44]. MiR-29s were found to inhibit Wnt/β-catenin signaling through demethylation of WIF-1 [45]. Upregulation of miR-182 and *HOXA9* silencing inhibited OS progression. We found that miR-182 downregulated Wnt/β-catenin signaling, inhibited cell proliferation, and promoted apoptosis in OS cells by suppressing *HOXA9* expression.

Reduced cell proliferation, percentage of cells in S phase, and tumor growth/volume, but an enhanced percentage of cells in G0/G1 and an increase in apoptosis was observed in the miR-182 mimic and siRNA-HOXA9 groups compared to the blank, NC, and miR-182 inhibitor + siRNA-HOXA9 groups. Opposite results were observed in the miR-182 inhibitor group. Centromeres are replicated during S phase of the cell cycle [46]. Cells in the G1 phase are more susceptible to differentiation [47]. Cell cycle arrest in G1 and an increase in apoptosis were observed in cells transfected with miR-182 [42]. MiR-182 was shown to induce cell cycle arrest by suppressing Survivin expression in tongue squamous cell carcinoma [48].

The article "MicroRNA-182 downregulates Wnt/β-catenin signaling, inhibits proliferation, and promotes apoptosis in human osteosarcoma cells by targeting HOXA9" was retracted in 2022. Reasons: fabricated or falsified data; manipulated images; an official misconduct investigation; misconduct by an author.

In conclusion, this study brings novel insight for the OS treatment in a molecular level, indicating that the miR-182 inhibiting Wnt/β-catenin signaling pathway can promote apoptosis but inhibit proliferation of human OS cells by suppressing HOXA9, meanwhile, provides a new biomarker for further study. The miRNAs dysregulation occurs frequently in various tumors and the utility of miRNAs in the preclinical stage is its infancy, but we can't afford to ignore that expanding exponentially as the enormous potential of these small molecules is becoming evident. The findings in this study provided underlying molecular mechanism for further investigation that upregulation of miR-182 and silencing of *HOXA9* can inhibit cell proliferation and enhance apoptosis in OS, suggesting that miRNAs have therapeutic potential and could also be novel prognostic markers. Activated Wnt/β-catenin signaling has been associated with tumorigenesis and metastasis and could be an early-stage diagnostic biomarker in OS.

## MATERIALS AND METHODS

### Ethical statement

This study was approved by the Ethics Committee of the Key Laboratory for Biotechnology on Medicinal Plants of Jiangsu Province, School of Life Science, Jiangsu Normal University. Written informed consent was obtained from all patients.

### Study subjects

Forty-six tumor tissue samples (the OS group) were obtained from patients with pathologically confirmed OS who underwent surgical resection at the Key Laboratory for Biotechnology on Medicinal Plants of Jiangsu Province, School of Life Science, Jiangsu Normal University between October 2011 and October, 2016. OS samples exhibited hardened textures. Lesions were found to arise from the periosteum, tumor periphery, and areas of trabecular destruction by X-ray. There were 27 male and 19 female patients. The average age was 25.59 ± 10.95 years (range, 11–65). An additional 46 normal bone tissue samples (the normal group) were collected from patients who underwent amputation. No significant differences in gender or age were observed between the normal and OS groups. Tissue samples were numbered, recorded, and stored at –80°C in liquid nitrogen. This study was approved by the Ethics Committee of the Key Laboratory for Biotechnology on Medicinal Plants of Jiangsu Province, School of Life Science, Jiangsu Normal University. Written informed consent was obtained from all patients.

The article "MicroRNA-182 downregulates Wnt/β-catenin signaling, inhibits proliferation, and promotes apoptosis in human osteosarcoma cells by targeting HOXA9" was retracted in 2022. Reasons: fabricated or falsified data; manipulated images; an official misconduct investigation; misconduct by an author.

### Immunohistochemistry

Tissue samples were fixed in 10% formaldehyde, embedded in paraffin, and sliced into 4 μm serial sections. Sections were dried in a 60°C incubator for 1 h, dewaxed in xylene (3 × 10 min), and then dehydrated in a graded series of alcohol (95%, 80%, and 75%, 1 min each). Sections were then washed with water for 1 min, incubated in 3% H_2_O_2_ at 37°C for 30 min, and washed with phosphate-buffered saline (PBS). Sections were boiled in 0.01 M citric acid buffer at 95°C for 20 min for antigen repair. After cooling to room temperature, sections were washed with PBS, blocked with normal goat serum at 37°C for 10 min, and incubated overnight with an anti-rabbit HOXA9 polyclonal antibody (ab191178, Abcam, Cambridge, MA, USA, 1:40 dilution) at 4°C. Following the incubation, sections were washed with PBS for 2 min and then incubated with a horseradish peroxidase (HRP)-conjugated secondary antibody (DF7852, Shanghai Yaoyun Biotechnology Co., Shanghai, China, 1:40 dilution) at room temperature for 30 min. Sections were then stained with diaminobenzidine (DAB, CAS: 7411-49-6, Suzhou Industrial Park for Subfamily Chemical Reagent Co., Ltd., Jiangsu, China). Sections were counterstained with hematoxylin (Shanghai Bogoo Biotech Company, Shandhai, China) and sealed. The primary antibody was replaced with PBS as a negative control. A total of 10 fields were selected for each section and 100 cells in each field were chosen randomly to count positive cells. Weakly positive cells were stained light yellow, moderately positive cells were brown/yellow, and strongly positive cells were brown [49].

### RT-qPCR

Total RNA was extracted from OS and normal tissue using the miRNeasy Mini Kit (217004, Qiagen, Hilden, Germany). Primers to amplify miR-182, *HOXA9*, *Wnt*, *β-catenin*, *WIF-1*, *Survivin*, *Cyclin D1*, *c-Myc*, *BIM*, *Bax*, *Mcl-1*, *Bcl-xL*, *Snail*, and U6 were designed and synthetized by the Takara Biotechnology Ltd. (Liaoning, China) (Table 1). Reverse transcription was performed with the PrimeScript RT Kit (RR036A, Takara Biotechnology Ltd., Liaoning, China) according to the manufacturer's protocol. The total reaction volume was 10 μL. The reaction conditions were as follows: reverse transcription at 37°C (15 min*3) and reverse transcriptase enzyme inactivation at 85°C for 5 s. RT-PCR was performed by SYBR^®^ Premix Ex Taq^TM^ II kit (RR820A, Takara Biotechnology Ltd., Liaoning, China). The reaction volume was 50 μL: 25 μL of SYBR^®^ Premix Ex Taq^TM^ II (2 ×), 2 μL forward primer, 2 μL reverse primer, l μL ROX Reference Dye (50 ×), 4 μL DNA template, and 16 μL ddH_2_O. RT-qPCR was performed with an ABI7500 instrument (7500, ABI Company, Oyster Bay, NY, USA). The reaction condition were as follows: pre-denaturation at 95°C for 30 s, 40 cycles of denaturation at 95°C for 30 s, annealing at 60°C for 30 s, and extension at 60°C for 30 s. U6 was used as an internal reference for miR-182 and *GAPDH* for *HOXA9*, *Wnt*, β-catenin, *WIF-1*, *Survivin*, *Cyclin D1*, *c-Myc*, *BIM*, *Bax*, *Mcl-1*, *Bcl-xL*, and *Snail*. Relative gene expression was calculated using the 2^-ΔΔCt^ method: ΔΔCt = ΔCt _(OS group)_ − ΔCt _(normal group),_ ΔCt = Ct _(target gene)_ − Ct _(internal reference)_ [50].

The article "MicroRNA-182 downregulates Wnt/β-catenin signaling, inhibits proliferation, and promotes apoptosis in human osteosarcoma cells by targeting HOXA9" was retracted in 2022. Reasons: fabricated or falsified data; manipulated images; an official misconduct investigation; misconduct by an author.

**Table 1:** The primer sequences for RT-qPCR

Primer	Sequence
miR-182	F: 5′-GGCAATGGTAGAACTCACACT-3′
	R: 5′-AACATGTACAGTCCATGGATG-3′
HOXA9	F: 5′-TGCCCTCCAGCCGGCCTTAT-3′
	R: 5′-CCGCTTTGTGCGGGGATGGT-3
Wnt	F: 5′-GCTAGCGAAAGTCATTGGC -3′
	R: 5′-CATTGCATCGAAGTCGTG-3′
CTNNB1	F: 5′-ACAAACTGTTTTGAAAATCCA-3′
	R: 5′-CGAGTCATTGCATACTGTCC-3′
WIF-1	F: 5′-CCGAAATGGAGGCTTTTGTA-3′
	R: 5′-TGGTTGAGCAGTTTGCTTTG-3′
Survivin	F: 5′-CCGAGGGACTGTGTGGGGGTC-3′
	R: 5′-CCAGGCACAGACCAAGGACGC-3′
CCND1	F: 5′-AATGGGCCTTAGAATGACTGC-3′
	R: 5′-ATGCCAACACAGATGGCTTT-3′
C-myc	F: 5′-CTACCAGCAGCAGCAGCAGAGC-3′
	R: 5′-CGTCCGGGTCGCACATGAA-3′
BIM	F: 5′-CGTAGCGCATGCGATA-3′
	R: 5′-CATGCCGTATAAGCTAGTT-3′
Bax	F: 5′-GGCCCACCAGCTCTGAGCAGA-3′
	R: 5′-GCCACGTGGGGGTCCCAAAGT-3′
Mcl-1	F: 5′-AGAAAGCTGCATCGAACCATTA-3′
	R: 5′-GGAAGAACAACTCCACAAACCCATC-3′
Bcl-xl	F: 5′-TTGGACAATGGACTGGTTGA-3′
	R: 5′-GTAGAGTGGATGGTCAGTG-3′
Snail	F: 5′-CTCCTCTACTTCAGCCTCTT-3′
	R: 5′-CTTCATCAACGTCCTGTGGG-3′
GAPDH	F: 5′-CCACCCATGGCAAATTCCATGGCA-3′
	R: 5′-TCTAGACGGCAGGTCAGGTCCAC-3′
U6	F: 5′-CTCGGCTTCGGCAGCACA-3′
	R: 5′-AACGCTTCACGAATTTGCGT-3′

Note: miR-182, microRNA-182; HOXA9, Homeobox A9; WIF-1, Wnt inhibitory factor-1; BIM, B-cell CLL/lymphoma-2 interacting mediator of cell death; Bcl, B-cell CLL/lymphoma; Mcl, Mantle cell lymphoma; RT-qPCR, reverse transcription-quantitative polymerase chain reaction; R, reverse; F, forward; GAPDH, Glyceraldehyde-3-phosphate dehydrogenase.

### Western blotting

Total protein was extracted from OS tissue using a RIPA kit (R0010, Beijing Solarbio Science & Technology Co., Ltd., Beijing, China). The total protein concentration was estimated using a BCA protein assay kit (69-21875, Wuhan Mokesha Biotech Company, Hubei, China). Proteins were separated by 10% SDS-PAGE (20050227, Beyotime Biotechnology Co., Shanghai, China) and transferred onto membranes. The membranes were incubated overnight at 4°C with HOXA9 (1: 2000, ab140631), Wnt (1: 3000, ab28472), β-catenin antibody (1: 5000, ab32572), WIF-1 (1: 2000, ab171766), Survivin (1: 10000, ab76424), Cyclin D1 (1: 10000, ab134175), c-Myc (1: 10000, ab166837), BIM (1:2000, ab32158), Bax (1: 2000, ab32503), Mcl-1 (1: 1000, ab32087), Bcl-xL (1: 2000, ab32503), or Snail (1: 500, ab53519) rabbit anti-human antibodies, which were purchased from Abcam (Cambridge, MA, USA). Membranes were then incubated with an HRP-conjugated goat anti-rabbit IgG secondary antibody (1: 1000, BA1056, Wuhan Boster Biological Technology Co., LTD., Hubei, China) or an HRP-conjugated goat anti-mouse IgG antibody (1: 5000; Zhongshan Biotech Ltd., Beijing, China). Blots were developed in the dark using the ECL reagent (WBKLS0500, Pierce, Rockford, IL, USA) and imaged.

The article "MicroRNA-182 downregulates Wnt/β-catenin signaling, inhibits proliferation, and promotes apoptosis in human osteosarcoma cells by targeting HOXA9" was retracted in 2022. Reasons: fabricated or falsified data; manipulated images; an official misconduct investigation; misconduct by an author.

### Dual-luciferase reporter assays

Dual-luciferase reporter assays were used to verify the targeting of the HOXA9 3′UTR by miR-182. The target sequence in the HOXA9 3′UTR was synthetized and inserted into the pMIR-REPORT vector between the SpeI and HindIII sites. The mutant site complementary to the seed region in HOXA9-wt was designed with the following primers: 5′-GCTCTAGATGCCATTTGGGCTTAT-3′ (forward) and 5′-TGCACTGCAG GGCTCCTATTTCCCTCTT-3′ (reverse). The target sequence was ligated into the pMIR-reporter vector using T4 DNA ligase. The HOXA9-wt and HOXA9-mut constructs were then cotransfected with miR-182 into human embryonic kidney (HEK)-293T cells (Shanghai Beinuo Biotech Ltd., Shanghai, China). Cells were collected and lysed 48 h after transfection. Luciferase activity was measured using a luciferase assay kit.

### Cell culture and transfection

SOSP-9607, U-2OS, MG63, and hFOB cells were purchased from the Shanghai Cell Center. Cells were seeded in RPMI-1640 media containing 10% fetal bovine serum (FBS) and mycillin and cultured in a 5% CO_2_ incubator at 37°C. The media was replaced every 24–48 h. Cells were digested with trypsin and passaged. Cells were used in experiments after three passages. Cell lines with relatively high miR-182 expression were identified using RT-qPCR. We divided the cells into blank, negative control (NC), miR-182 mimics, miR-182 inhibitor, siRNA-HOXA9, and miR-182 inhibitor + siRNA-HOXA9 groups. Cells were seeded into 6-well plates 24 h before transfection. When the cells reached approximately 50% confluence, they were transfected using Lipofectamine 2000 (11668027, Invitrogen Inc., Carlsbad, CA, USA). Plasmids (NC, miR-182 mimics, miR-182 inhibitor, siRNA-HOXA9, and miR-182 inhibitor + siRNA-HOXA9, 100 pmol) were diluted in serum-free Opti-MEM (250 μl, 31985-070, Gibco, Grand Island, NY, USA) to a final concentration of 50 nM, mixed, and incubated at room temperature for 5 min. We diluted 5 μl of Lipofectamine 2000 in 250 μL serum-free Opti-MEM and incubated the mixture at the room temperature for 5 min. Next, the diluted plasmid solution containing cells was mixed with Lipofectamine 2000 and the cells incubated at room temperature for 20 min. Following the incubation, cells were seeded into plates and cultured at 37°C with 5% CO_2_ for 6–8 h. The media was then replaced with complete media. Cells were used in experiments after 24–48 h.

The article "MicroRNA-182 downregulates Wnt/β-catenin signaling, inhibits proliferation, and promotes apoptosis in human osteosarcoma cells by targeting HOXA9" was retracted in 2022. Reasons: fabricated or falsified data; manipulated images; an official misconduct investigation; misconduct by an author.

### CCK-8 assays

Once hFOB and USOS cells reached 80% confluence (approximately 12 h after transfection), they were washed twice with PBS and digested with 0.25% trypsin to prepare single cell suspensions. Cells were counted and 3 × 10^3^–6 × 10^3^ cells seeded into each well (200 μL, six parallel wells) of a 96-well plate and incubated at 37°C. We then added 10 μL of CCK-8 (Sigma-Aldrich Chemical Company, St Louis MO, USA) to each well 24, 48, or 72 h after seeding. Following a 2 h incubation, the optical density of each well was measured at 450 nm using enzyme-linked immunosorbent instrument (NYW-96M, Beijing Noah Instrument Co., Ltd., Beijing, China). Experiments were repeated three times.

### Flow cytometry

PI staining was used to detect cell cycle phase. Cells were collected and fixed in 70% ice-cold ethanol overnight at 4°C. Cells were then centrifuged at 4°C and the supernatants discarded. Cells were washed twice with PBS containing 1% FBS, resuspended in 400 μL binding buffer, and incubated with 50 μL RNase (Sigma-Aldrich, St. Louis MO, USA) at 37°C for 30 min. Finally, cells were stained with 50 μL 50 mg/L PI (Sigma-Aldrich) for 30 min at room temperature in the dark. Cell cycle phase was detected by flow cytometry.

Apoptosis was analyzed using the Annexin-V/PI double labeling method. Cells were digested with 0.25% trypsin without EDTA (YB15050057, Shanghai Yubo Biological Technology Co., Ltd, Shanghai, China) 48 h after transfection, centrifuged, and the supernatants discarded. The cell pellets were washed three times with cold PBS and the supernatants discarded. Annexin-V-FITC/PI staining was performed using the Annexin-V-FITC Apoptosis Kit (K201-100, BioVision, CA, USA) and the manufacturer's instructions. The Annexin-V-FITC/PI staining solution was prepared by mixing Annexin-V-FITC, PI, and HEPES buffer at a 1: 2: 50 ratio, respectively. We added 100 μL of the staining solution to 1 × 10^6^ cells, incubated the cells at room temperature for 15 min, and then added 1 mL of HEPES buffer (PB180325, Procell, Hubei, China). Cell fluorescence was measured using a 620 nm bandpass filter for PI and a 525 nm bandpass filter for FITC after excitation at 488 nm, and apoptosis quantified. Experiments were repeated three times.

The article "MicroRNA-182 downregulates Wnt/β-catenin signaling, inhibits proliferation, and promotes apoptosis in human osteosarcoma cells by targeting HOXA9" was retracted in 2022. Reasons: fabricated or falsified data; manipulated images; an official misconduct investigation; misconduct by an author.

### Wound healing assays

Cells were seeded in the plate 12 h after transfection at a density of 40%. After 24 h, cell monolayers were wounded by scratching using a sterile 200 μL pipette tip. Cells were then rinsed twice with PBS to remove debris, and cultured in serum-free medium. Images of the wounds were acquired at 0 h and 48 h. Cell migration was quantified by analyzing the degree of wound closure.

### Xenograft tumors in nude mice

Human OS cells were resuspended in a mixture of PBS/Matrigel (1: 1 v/v) at a final cell concentration of 1 × 10^6^/200 μL. Eighteen nude mice were divided into blank, NC, miR-182 mimic, miR-182 inhibitor, siRNA-HOXA9, and miR-182 inhibitor + siRNA-HOXA9 group (three mice per group). Nude mice were anaesthetized using diethyl ether and inoculated with 1 × 10^6^ OS cells (per 200 μL). The mice were fed under the same conditions. Tumor lengths and widths were recorded once a week and tumor volume calculated using the following formula: volume = (length × width^2^)/2. Mice were sacrificed 35 days after inoculation. Three tumors were collected from each group.

### Statistical analysis

Statistical analysis was performed using the SPSS 21.0 software (IBM Corp., Armonk, NY, USA). Data are presented as the mean ± standard deviation. Comparisons between two groups were analyzed using *t*-tests. Comparisons among multiple groups were assessed using one-way analysis of variance. A *P* < 0.05 was considered statistically significant.
